The article "Overexpression of Mineralocorticoid Receptors in the Mouse Forebrain Partly Alleviates the Effects of Chronic Early Life Stress on Spatial Memory, Neurogenesis and Synaptic Function in the Dentate Gyrus" was published in 2017. Journal: Front Cell Neurosci.

# Overexpression of Mineralocorticoid Receptors in the Mouse Forebrain Partly Alleviates the Effects of Chronic Early Life Stress on Spatial Memory, Neurogenesis and Synaptic Function in the Dentate Gyrus

**DOI:** 10.3389/fncel.2017.00132

**Published:** 2017-05-29

**Authors:** Sofia Kanatsou, Henk Karst, Despoina Kortesidou, Rachelle A. van den Akker, Jan den Blaauwen, Anjanette P. Harris, Jonathan R. Seckl, Harm J. Krugers, Marian Joels

**Affiliations:** ^1^Department of Translational Neuroscience, Brain Center Rudolf Magnus, University Medical Center UtrechtUtrecht, Netherlands; ^2^Swammerdam Institute for Life Sciences – Center for Neuroscience, University of AmsterdamAmsterdam, Netherlands; ^3^Endocrinology Unit, Centre for Cardiovascular Science, Queen’s Medical Research Institute, The University of EdinburghEdinburgh, United Kingdom; ^4^University of Groningen, University Medical Center GroningenGroningen, Netherlands

**Keywords:** mineralocorticoid receptor, early life stress, mouse, hippocampus, spatial memory, synaptic transmission, neurogenesis, electrophysiology

## Abstract

Evidence from human studies suggests that high expression of brain mineralocorticoid receptors (MR) may promote resilience against negative consequences of stress exposure, including childhood trauma. We examined, in mice, whether brain MR overexpression can alleviate the effects of chronic early life stress (ELS) on contextual memory formation under low and high stress conditions, and neurogenesis and synaptic function of dentate gyrus granular cells. Male mice were exposed to ELS by housing the dam with limited nesting and bedding material from postnatal day (PND) 2 to 9. We investigated the moderating role of MRs by using forebrain-specific transgenic MR overexpression (MR-tg) mice. Low-stress contextual (i.e., object relocation) memory formation was hampered by ELS in wildtype but not MR-tg mice. Anxiety like behavior and high-stress contextual (i.e., fear) memory formation were unaffected by ELS and/or MR expression level. At the cellular level, an interaction effect was observed between ELS and MR overexpression on the number of doublecortin-positive cells, with a significant difference between the wildtype ELS and MR-tg ELS groups. No interaction was found regarding Ki-67 and BrdU staining. A significant interaction between ELS and MR expression was further observed with regard to mEPSCs and mIPSC frequency. The ratio of evoked EPSC/IPSC or NMDA/AMPA responses was unaffected. Overall, these results suggest that ELS affects contextual memory formation under low stress conditions as well as neurogenesis and synaptic transmission in dentate granule cells, an effect that can be alleviated by MR-overexpression.

## Introduction

Environmental factors in interaction with the genetic background of individuals determine the vulnerability or resilience to subsequent stress-related psychopathology (Caspi et al., 2003). One of such important environmental risk factors for the later development of e.g., depression and post-traumatic stress disorder is early life adversity, particularly in vulnerable individuals (Caspi et al., 2003; Klengel et al., 2013).

The effects of early life adversity may be mediated by long-lasting alterations in the regulation of the hypothalamus-pituitary-adrenal (HPA)-axis and stress responsiveness. Exposure to stress increases the release of glucocorticoid hormones (cortisol in humans; corticosterone in rodents) from the adrenal glands (de Kloet et al., 2005). Glucocorticoids bind to high-affinity mineralocorticoid receptors (MRs) and lower-affinity glucocorticoid receptors (GRs). Activation of MRs and GRs alter brain cell function via both non-genomic and genomic mechanisms (Joëls et al., 2012) ultimately promoting behavioral adaptation to stressful conditions (de Kloet et al., 1999; Schwabe et al., 2010). However, early life adversity may program the release of glucocorticoids and other aspects of the HPA-function for the rest of the lifespan (Sapolsky and Meaney, 1986; Ivy et al., 2008). The mechanism by which early life effects are exerted appears to involve epigenetic modifications of MR and GR gene promoters (Szyf et al., 2005; Heim and Binder, 2012) notably in limbic regions such as the hippocampus. The consequent persistent alterations in hippocampal MR and GR density may contribute to altered vulnerability to psychopathology (Klengel et al., 2013).

In humans, polymorphisms of the MR-encoding gene NR3C2 (notably the MR-I180V single-nucleotide polymorphism) reduce MR function and have been associated with increased prevalence of depressive symptoms (Kuningas et al., 2007; Klok et al., 2011a). Conversely, a common MR haplotype, resulting *in vitro* in increased MR expression and functionality, is associated with a heightened dispositional optimism and lower depression scores in the face of multiple life events, at least in women (Klok et al., 2011b; Vinkers et al., 2015). In rodents, activation of MRs prevents granular cells from apoptosis (Sloviter et al., 1989) and facilitates long-term potentiation (Pavlides et al., 1994). In addition, we have recently reported that increased MR functionality may protect against the consequences of chronic stress exposure (Kanatsou et al., 2015a).

The aim of the current study was to examine the potential causality between enhanced MR activity and resilience to early life adversity. Therefore we investigated, in mice, whether transgenic overexpression of MRs (Lai et al., 2007) is able to protect against earlier reported (Brunson et al., 2005; Rice et al., 2008; Naninck et al., 2015) adverse effects of chronic early life stress on cognitive function and relevant cellular endpoints for memory formation.

## Materials and Methods

### Animals and Breeding Procedure

Animals were kept under standard housing conditions (12 h light/dark cycle, lights on at 8:00 a.m., humidity 40–60%, temperature 21.5 – 22°C) with *ad libitum* access to food and water. All experiments were performed in strict accordance with the Dutch regulations for animal experiments. The protocol was approved by the committee on Animal Health and Care of University of Amsterdam, the Netherlands (permit number DED 291).

For all experiments, heterozygous animals with forebrain MR overexpression (MR-tg), generated by inserting the HA-tagged human MR cDNA using the CaMKIIα promoter (MR-tg animals, Lai et al., 2007) and control littermates mice were generated in-house as reported previously (Kanatsou et al., 2015a,b). Because of the CaMKII promoter, MR overexpression did not take place until the end of the second postnatal week (J. R. Seckl, personal communication). Pregnant (wildtype) females were single housed at the beginning of the third gestational week and monitored daily for birth (9:00 a.m.). To minimize unnecessary stress we left the cages – that were covered with filter-tops until weaning -with the pregnant females in a separate breeding room. When a litter was found at 9:00 a.m., we assigned the day before as the day of birth (PND0).

### Early Life Stress Paradigm

To introduce a period of chronic early life stress, we used a model of fragmented maternal care that has previously been reported in mice (Rice et al., 2008; Wang et al., 2011; Baram et al., 2012; Naninck et al., 2015; Arp et al., 2016; Lesuis et al., 2016). Therefore dams with pups were housed with limited nesting and bedding material (ELS) from Postnatal Day (PND2-PND9). On the morning of PND2 we recorded the bodyweight of the mothers and the pups and culled the litter size to 6 pups (including both genders). We then randomly assigned the dams and pups to either the ELS or control condition. In the control situation, dams were provided with a standard amount of sawdust bedding and nesting material (one square piece of cotton nesting material (5 × 5 cm; Technilab-BMI, Someren, The Netherlands). ELS was induced by housing the dams in a cage with a fine-gauge stainless steel mesh that was placed 1 cm above the cage floor. The bottom was covered with reduced amount of sawdust bedding and nesting material (1/2 square piece of cotton nesting material, Technilab-BMI, Someren, The Netherlands). From PND2-PND9 the cages were left undisturbed. At PND9, we weighed both the dams and their litters and transferred them together to cages with a normal amount of sawdust bedding and nesting material until weaning. The cages were then refreshed once per week until weaning (PND23). Upon weaning, we recorded the bodyweight of the dams and the pups and we collected ear tissue for genotyping. All experiments described here were performed in male mice. One week after weaning, we housed male mice coming from a different dam two per cage to avoid litter effects. All experimental cages were covered with filter-tops and refreshment of the cages occurred once per week with no extra manipulation that could affect the mice.

### Behavior

Behavioral testing occurred in 4 months’ old mice during the light phase (9:00 a.m. -13:00 a.m.). Mice were tested for anxiety-like behavior and learning and memory. To assess learning and memory, we used behavioral tests with low levels of arousal (object in-context task, object location task; Kanatsou et al., 2015a,b) and tests with high levels of arousal (contextual fear conditioning and extinction). Two different cohorts of animals were used for behavioral testing: one cohort was tested in the open field, the object in context task and the object location task (5 days interval in between each behavior test). A second cohort was used for contextual fear conditioning to avoid confounding effects of previous testing. Data obtained from the open field were analyzed with an EthoVision video tracking system. The same experimenter, blinded to the treatment and genotype, analyzed all other behavioral data manually using video recordings.

#### Open Field

The open field paradigm we used is part of the protocol of the object in-context paradigm. On the first day of the protocol, animals were exposure to an open field (arena, W × L × H; 33 cm × 54 cm × 37 cm) and were allowed to freely explore for 10 min. Mice were facing the same wall when introduced in the arena and we refreshed the bedding material covering the bottom with new bedding material between the different animals. After testing, the mouse was removed from the arena and brought back to its home cage. To assess anxiety-like behavior we used the total time that the mice spent in the central area of the arena. For locomotor activity we used the total distance the mice spent in the arena for the total 10 min of exploration. The analysis was performed using the Ethovision XT 6 (Noldus, Wageningen, The Netherlands).

#### Object in Context Recognition Memory

To assess contextual memory, we used the object in context task (Ennaceur and Aggleton, 1997; Bussey et al., 1999; Mumby et al., 2002; Stupien et al., 2003; Winters et al., 2004; Balderas et al., 2008; Kanatsou et al., 2015a,b) that is based on the classical object-context novelty preference paradigm (Dix and Aggleton, 1999). The protocol consists of 3 days; a habituation phase, a training phase and the testing phase. On day 1 (habituation) mice were placed in an arena (plastic box, W × L × H; 33 cm × 54 cm × 37 cm) and were allowed to explore the context for 10 min (for more details see above open field). During the training phase, mice were exposed to two different contexts. In context A (plastic box without cues, W × L × H; 33 cm × 54 cm × 37 cm) the mouse was allowed to explore a set of similar objects (Lego blocks) for 10 min. Immediately after testing the mouse was placed back in its transfer cage and after 1 min retention we trained the mouse in context B. Context B had the same size of context A but it was different since it had cues on all walls and contained a different set of objects (glass bottles). The mouse was allowed to explore this arena for 10 min and after training it was returned back to its home cage. During training, mice were placed in the contexts by facing the wall opposite to the objects. All objects were cleaned thoroughly between tests with 70% ethanol and the bedding material that covered the bottom was refreshed with new one and mixed thoroughly, between each trial.

To examine recognition memory, mice were placed back in context B for 10 min during the testing phase (on day 3) with one bottle (familiar object) and one Lego-object (novel object for this context) present. The context discrimination index (DI) was calculated as: (the time mice spent with the novel object in context B)/(time of exploration of familiar object in context B + time of exploration of novel object in context B) (Akkerman et al., 2012). An index > 0.5 reflects recognition memory of the novel object in relation to the context (Lego in context B). We defined ‘sniffing behavior’ as the mouse with its nose being within 2 cm of the object. Climbing on top of the objects was not considered as sniffing behavior.

#### Object Relocation Memory

We used the object relocation memory test (OLT) to test place memory in mice (Luine et al., 2003). On day 1, mice were habituated to an arena (W × L × H; 23,5 cm × 31 cm, height × 27 cm) for 5 min and were then placed back to their home cage. On day 2 of the protocol, mice were trained for 5 min in the arena with a set of similar objects (set of glass cups) that were placed 12 cm from each other and 11 cm from the wall. On day 3 (testing day), we moved one of the objects in a novel location and mice were exploring for 5 min.

All arenas used were covered with sawdust bedding that was refreshed with new one in between trials. All objects were cleaned with 25% ethanol. To assess spatial memory, we used the DI as mentioned above.

#### Contextual Fear Conditioning and Extinction

To examine fear memory we used a contextual fear-conditioning paradigm. The apparatus consisted of a chamber (W × L × H: 25 cm × 25 cm × 30 cm) with cues on the wall and was equipped with a stainless steel grid floor connected to a shock generator (Zhou et al., 2009, 2010; Kanatsou et al., 2015a,b).

During training (day 1), mice were introduced in the chamber and habituated for 3 min followed by a single foot shock (0.4 mA for 2 s). On day 2 (contextual fear memory), mice were placed back in the same chamber and were allowed to explore the context for 3 min. On day 3 and day 4, we repeated the same procedure for 3 min to monitor extinction of learned behavior. The chamber was cleaned with 70% ethanol between testing. We used freezing behavior as an index of fear memory. Freezing was defined as no body movement except those required for respiration (Maren, 2001; Zhou et al., 2009) and was expressed as percentage of total time.

### Neurogenesis

To study the long-term effect of ELS on the different stages of adult hippocampal neurogenesis, we administered intraperitoneally a total dose of 300 mg/kg BrdU ((Sigma–Aldrich, St. Louis, MO, United States) 10 mg/ml in 0.007 M NaOH/0.9% NaCl) via three injections of 100 mg/kg with an interval of 2 h between each injection in 3 months’ old mice (a different set of animals than those tested for behavior) (Oomen et al., 2007; Hu et al., 2012; Kanatsou et al., 2015a). When mice were 4 months’ old, they were anesthetized with Euthasol (120 mg/kg; Produlab Pharma, the Netherlands) and transcardially perfused with a paraformaldehyde solution (4% paraformaldehyde in 0.1M phosphate buffer pH7.4). To prevent pressure artifacts, the brains were extracted carefully, post-fixed for 24 h at 4°C in paraformaldehyde and cryoprotected by sucrose solution (30% sucrose in 0.1 M phosphate buffer, pH7.4) on a shaking platform at 4°C. Brains were cut into 40 μm thick sections using a sliding microtome, collected in antifreeze solution (30% Ethylene glycol, 20% Glycerol, 50% 0,05M PBS) and stored at -20°C.

To study the different stages of the neurogenesis process (Mayer et al., 2006), we performed immunohistochemistry. To assess the 4 weeks’ survival of newborn cells, we incubated the sections overnight at 4°C with a primary antibody [rat monoclonal anti-Bromodeoxyuridine antibody, 1:500, CloneBU1/75 (ICR1), Accurate Chemical, country] (Marlatt et al., 2010; Naninck et al., 2015). To assess proliferation at the time of tissue collection, we used the rabbit polyclonal anti-Ki-67 antibody (1:10000, NCL-L-Ki67_MM1, Novocastra, Newcastle upon Tyne, United Kingdom) (Marlatt et al., 2010). Doublecortin (DCX) (polyclonal goat anti-DCX, 1:800, sc-8066, Santa Cruz, Leiden, the Netherlands) was assessed to examine the maturation of newborn cells (Marlatt et al., 2010). Sections were washed with 0.05M TBS for 2 h on a shaking platform at room temperature with secondary antibodies (biotinylated sheep anti-mouse 1:200 (GE Healthcare, United Kingdom), goat anti-rabbit 1:200 (Vector Laboratories, Burlingame, CA, United States) or biotinylated donkey anti-goat 1:500 (kindly provided by Dr. I. Huitinga, Netherland Institute for Neuroscience, Amsterdam) and for 90 min with avidin-biotin (ABC kit, 1:800, Elite Vectastain, Brunschwig Chemie, Amsterdam, the Netherlands). Sections were washed in 0.05 M Tris-buffer (TB), pH7.4 and subsequently chromogen development was performed for 6 min with diaminobenzidine (DAB) (20 mg per 100 ml of Tris buffer, 0.01% H2O2).

For quantification, sections that were folded, broken or had uneven staining were not selected for analysis. The cells stained for BrdU, DCX and Ki67 were counted bilaterally along the rostral-caudal hippocampal axis using a light microscope (40x objective, Zeiss) (Kanatsou et al., 2015a). The sum of the counted cells was multiplied by six (each brain was sectioned coronally in six parallel series) to calculate the total number of stained neurons in the dentate gyrus (DG; Kanatsou et al., 2015a). As the density of DCX+ cells was too high to count manually, this was counted using an automated stereology program, performed with the StereoInvestigator system (Microbrightfield, Germany). Contours were drawn for each hippocampal section and the cells were counted using an optical fractionator at 40x magnification (Axiophot, Zeiss-West Germany). Optical fractionator settings were 70 × 80 counting grid size and 25 × 25 counting frame size.

Neurogenesis was measured in the entire DG and also along both the suprapyramidal blade and the infrapyramidal blade of the hippocampus. This is relevant since neurogenesis is not homogeneous in both blades and these blades may have distinct behavioral functions (Olariu et al., 2007; Sahay and Hen, 2007; Snyder et al., 2009). Based on the bregma points of the sections, we further made a distinction between the numbers of cells found in the rostral and caudal part respectively of the DG. Due to the curvature of the hippocampus, it is difficult to make an accurate distinction between the rostral and caudal subareas of the hippocampus (Functional Neurogenesis website. Accessed October 11, 2012). Therefore, sections with bregma -1.34 to -2.70 were defined as the rostral DG while the sections between bregma point -2.80 to -3.80 were defined as the caudal part of the DG (Franklin and Paxinos, 1997). To correct for the variation in the amount of sections between the animals, seven sections per animal were selected.

### Electrophysiology

In a different set of animals, electrophysiological properties were determined in granular cells of the dorsal hippocampal DG. At the day of the electrophysiological experiments, the mice were decapitated around 9 a.m. when plasma corticosterone levels are low. The brain was removed from the skull and stored in ice-cold artificial cerebrospinal fluid (ACSF) containing choline chloride instead of sodium chloride and low calcium and high magnesium of the following composition (in mM): 120 Choline Cl, 3.5 KCl, 1.25 NaH2PO4, 6.0 MgSO4, 0.5 CaCl, 25 NaHCO3, and 10 glucose; pH 7.4 gassed with 95% O_2_-5% CO_2_. In the same ACSF, horizontal slices of the brain were made with a vibratome (Campden Instruments, Sileby, United Kingdom). The slices containing the hippocampus were stored for 20 min in continuously gassed (95% O_2_-5% CO_2_) normal ACSF of 32°C containing (in mM): 124 NaCl, 3.5 KCl, 1.25 NaH2PO4, 1.5 MgSO4, 2 CaCl, 25 NaHCO3, and 10 glucose; pH 7.4. Next the slices were allowed to recover for >1 h in normal ACSF at room temperature.

#### Recording Evoked Currents

One slice at a time was placed in a recording chamber mounted on an upright microscope (Zeiss Axioskop), continuously perfused with normal ACSF (32°C, 2–3 ml/s) and kept fully submerged. Patch-clamp electrodes for recording (0.86 mm inner diameter, 1.5 mm outer diameter, borosilicate glass (Harvard Apparatus); impedance approximately 3–5 MΩ) were pulled on a Sutter (United States) micropipette puller and placed above the slice. The intracellular pipette solution contained (in mM): 120 Cs methane sulfonate, 17.5 CsCl, 10 Hepes, 2 MgATP, 0.1 NaGTP, 5 BAPTA, and 5 QX-314; pH 7.4, adjusted with CsOH. BAPTA was obtained from Molecular Probes (Leiden, The Netherlands); the sodium channel blocker QX-314 was from Alomone (Jerusalem, Israel). Under visual control (40x objective and 10x ocular magnification) the electrode was directed toward a granule neuron in the superficial blade of the DG using positive pressure. Once a patch electrode was sealed on the cell (resistance > 1 GΩ) the membrane patch under the electrode was ruptured and the cell was held at a holding potential of -65 mV. Signals were fed via a Digidata (1200 Axon Instruments) interface into an Axopatch 200B amplifier (Axon Instruments). Data acquisition and analysis was performed with PClamp (version 9.2).

A concentric bipolar stainless steel stimulus electrode (FHC, CBBRC75, outer diameter 200 μm, inner diameter 25 μm) was placed in the perforant path. Biphasic stimuli (250 μs) were applied through a Neurolog stimulus isolator (NL 800) driven by a Pclamp. Input–output curves of excitatory postsynaptic currents (EPSCs) evoked in DG neurons were made at holding potential by increasing stimulus intensities from 0 to 4 mA, given once every 10 s. EPSCs were recorded with a sampling frequency of 10 kHz. Signals were stored and analyzed off-line. Input–output curves were fit with a Boltzmann equation,

$$\begin{array}{c} R(i)\;=\;R_{\max}/[1\;+\;\exp\{(i\;-\;i_{H}){/I}_{C}\}], \end{array}$$

in which R_max_ is the maximal evoked current, i_H_ the half-maximal stimulus intensity, and I_C_ proportional to the slope. Based on this curve the half-maximal stimulus intensity was determined. This intensity was used to evoke 5 sweeps of evoked (e)EPSCs at a holding potential of -65 mV, i.e., the reversal potential of GABA currents, using intervals of 10 s. The averaged signal was used to determine the peak amplitude of the evoked EPSC mediated by AMPA receptors. Then the holding potential was set at the reversal potential for the glutamate currents at +10 mV and 5 sweeps at the half maximal intensity were delivered to determine the amplitude of synaptically evoked (e)IPSCs via GABA receptors. Subsequently we switched to a perfusion solution containing normal ACSF with bicuculline methiodide (20 μM, Sigma) to block the GABA-currents and stepped to a holding potential of +50 mV. At this holding potential both AMPA and NMDA currents are evoked, which can be distinguished based on their different inactivation properties (Karst and Joëls, 2003). At 150 ms after the onset of the evoked current the amplitude of the current exclusively contains evoked EPSCs mediated by NMDA receptors. Again 5 sweeps were averaged to determine the amplitude of the NMDA currents at half maximal stimulus intensity. The AMPA/NMDA ratio was calculated from the amplitudes of the AMPA and NMDA currents obtained at -65 and +50 mV respectively.

#### Recording Miniature Currents

To record the miniature (m)EPSCs and mIPSCs, another slice was placed in the recording chamber and perfused with normal ACSF at 32°C containing TTX (0.5 μM Latoxan) to block spontaneous spiking of the dentate neurons. A whole cell patch clamp recording was obtained as described above with the same internal pipette solution but without QX-314: (in mM) 120 Cs methane sulfonate, 17.5 CsCl, 10 Hepes, 2 MgATP, 0.1 NaGTP and 5 BAPTA; pH 7.4, adjusted with CsOH. When the recording was stable, recordings with a sampling frequency of 10 kHz at various holding potentials (see below) and a duration of 5 min were stored. At a holding potential of -65 mV, i.e., at the reversal potential of the GABA currents, AMPA receptor-mediated mEPCs were obtained. Subsequently, at the reversal potential of glutamate at +10 mV, GABA receptor-mediated mIPSCs were recorded. Data storage and acquisition was carried out with PClamp (version 9.2). Currents were identified as mEPSCs or mIPSCs when the rise time was faster than the decay time. The mEPSC and mIPSC amplitudes and frequency were determined and compared among the experimental groups.

### Statistical Analysis

Statistical analyses were performed using SPSS for Windows v17.0. Memory in the object-in-context and object relocation task was first tested for deviation from chance level (0.5) with a paired *t*-test. We applied an unpaired two-tailed Student’s *t*-test to assess the effect of ELS on bodyweight gain during the ELS paradigm. For all other analyses (where no time-effect was present) a two-way ANOVA was used to analyze the data, with ELS as the predicting factor and genotype as the moderating factor. When a time effect was present (e.g., with absolute body weight over time or in the fear memory extinction experiment) we used repeated-measures ANOVA over the different days of testing with “testing day” as the within-subjects factor and “genotype” and “treatment (ELS)” as fixed between-subject factors.

Huynh-Feldt correction was used to correct for violations of sphericity. Given our hypothesis we were primarily interested in significant interaction effects. These were followed up by *post hoc* comparisons with Fisher’s least significant difference (LSD). To correct for multiple comparisons (four meaningful comparisons) the alpha was set to be significant at *p* ≤ 0.0125 (^∗^) and 0.0125 < *p* ≤ 0.05 was considered to be a trend. All data are expressed as mean with standard error of the mean (SEM).

## Results

### Body Weight

First we examined the effectiveness of the limited nesting and bedding material model to induce ELS. Therefore we measured bodyweight, as previous studies have shown that this model reduces bodyweight gain at PND9 (Rice et al., 2008; Naninck et al., 2015). Pups exposed to ELS gained significantly less bodyweight from PND2-PND9 when compared to non-ELS controls [*t*(46) = 15.42, *p* < 0.001; **Figure 1A**] as described before (Rice et al., 2008), thereby supporting that the ELS procedure was effective in eliciting stress for the offspring. After PND9, body weight increased with age (main effect of time; *F*(2,70) = 1435.666, *p* < 0.001, **Figure 1B**). There was no persisting effect of ELS on body weight [*F*(2,70) = 2.107, *p* = 0.150] and no interaction between ELS and genotype on body weight [*F*(2,70) = 1.365, *p* = 0.257]. Yet, there was a significant interaction between age and genotype [*F*(2,70) = 15.485, *p* < 0.001], with MR-tg mice showing a significantly larger increase in body weight from PND23 to PND39 and from PND39 to PND120 (*p* < 0.001).

**FIGURE 1:** **Effect of ELS on bodyweight. (A)** Body weight gain during the period of ELS (PND2-PND9, *n* = 23–25) and **(B)** at discrete time points; upon weaning (PND23), at PND39 and at PND120 (initiation of behavioral testing). Data are expressed as mean ± SEM with *p*-values based on *post hoc* LSD. *n* = 7–12 mice per group. ^∗^Significant, *p* < 0.05.

### Behavior

#### Object In-context Recognition Memory

Stress exposure is known to enhance memory for fearful situations but impair memory when tested under less arousing conditions (McGaugh and Izquierdo, 2000). We therefore tested the animals in an object-in-location memory task that probes hippocampal function under non-arousing circumstances (Barsegyan et al., 2014). During testing on day 3, wildtype control mice demonstrated significant discrimination between the familiar and novel objects, since the DI was significantly higher than 50% (chance level). This was also the case for MR-tg mice with or without ELS, but not for wildtype mice exposed to ELS. There was a significant main effect of ELS [*F*(1,43) = 5.724, *p* = 0.022, **Figure 2A**] indicating that object in context learning did not occur in ELS animals. However, we did not find a significant interaction effect between genotype and ELS [*F*(1,43) = 1.165, *p* = 0.287].

**FIGURE 2:** **Recognition memory in MR-tg and control mice.** The discrimination index as observed in mice tested in **(A)** the object in-context task and **(B)** in object relocation task. Data are expressed as mean ± SEM with *p*-values based on *post hoc* LSD. *n* = 10–12 mice per group. ^∗^Significant, *p* ≤ 0.0125.

#### Object Relocation Memory

Mineralocorticoid receptors antagonists and genetic deletion of MRs have been shown to impair spatial memory (Oitzl and de Kloet, 1992; Yau et al., 1999; Berger et al., 2006). To assess whether MR overexpression modulates the effect of ELS, mice were tested in a spatial orientation task (i.e., the object relocation task). Overall, there was a significant interaction between genotype and ELS [*F*(1,43) = 11.507, *p* < 0.002, **Figure 2B**] and a significant main effect of ELS [*F*(1,43) = 48.723, *p* < 0.001] on contextual memory. *Post hoc* analysis revealed that ELS significantly reduced contextual memory in wildtype (*p* < 0.001) but not in MR-tg mice; MR-tg mice exposed to ELS outperformed wildtype animals exposed to ELS (*p* < 0.001).

#### Open Field Test

Pharmacological studies have reported that MRs affect anxiety-like behavior (Smythe et al., 1997; Bitran et al., 1998). We therefore tested all experimental groups in the open field test to measure their anxiety-like behavioral state. There was no main effect of ELS [*F*(1,43) = 3.025, *p* = 0.090], genotype [*F*(1,43) = 3.842, *p* = 0.057] nor any interaction of these two factors [*F*(1,43) = 2.519, *p* = 0.121] on the total distance mice traveled, suggesting that exploratory behavior and locomotion were not affected (**Figure 3A**). In terms of the total time that mice spent in the central area (**Figure 3B**), there was also no effect of ELS [*F*(1,43) = 1.146, *p* = 0.291], genotype [*F*(1,43) = 1.539, *p* = 0.222] nor any interaction [*F*(1,43) = 0.896, *p* = 0.350], indicating that this measure of anxiety-like behavior was unaffected by ELS or MR-tg.

**FIGURE 3:** **Open field behavior in MR-tg and control mice.** Bar graphs represent the results for **(A)** locomotion and **(B)** ‘anxiety-like behavior’ as measured by the total time mice spent in the central zone in the open field. Data are expressed as mean ± SEM. *n* = 10–12 mice per group.

#### Contextual Fear Conditioning and Extinction

To assess whether MR-overexpression –with or without prior exposure to ELS- affects memory in a high-arousing learning task we tested mice in a contextual fear conditioning task. During training (day 1) (**Figure 4**), mice were allowed to explore the chamber for 3 min before the foot shock was delivered. Analysis of freezing behavior before the foot shock showed neither a main effect of ELS [*F*(1,38) = 0.185, *p* = 0.670], genotype [*F*(1,38) = 0.641, *p* = 0.429] nor an interaction between genotype and treatment [*F*(1,38) = 0.115, *p* = 0.736]. Freezing behavior immediately after the foot shock also showed no main effect of ELS [*F*(1,38) = 1.840, *p* = 0.184], genotype [*F*(1,38) = 0.208, *p* = 0.651] nor an interaction [*F*(1,38) = 0.016, *p* = 0.900]. Also, freezing behavior during consolidation (day 2, i.e., re-exposure to the same context, **Figure 4**) revealed no significant effect of ELS [*F*(1,38) = 1.114, *p* = 0.299], genotype [*F*(1,38) = 1.479, *p* = 0.232] or an interaction effect [*F*(1,38) = 1.008, *p* = 0.322]. Finally, repeating the trails during days 3 and 4 revealed no significant extinction effect [repeated measures ANOVA, *F*(2,68) = 0.311, *p* = 0.727; **Figure 4**] nor a significant interaction effect of day, ELS and genotype [repeated measures ANOVA, *F*(2,68) = 1.470, *p* = 0.238].

**FIGURE 4:** **Contextual fear conditioning in MR-tg and control mice.** Bar graphs represent freezing time before the foot-shock (day 1), immediately after the foot-shock (day 1), and on day 2, day 3 and day 4. Data are expressed as mean ± SEM with *p*-values based on *post hoc* LSD. *n* = 8–11 mice per group.

### Neurogenesis

Neurogenesis has been implicated in cognition, fear and behavioral flexibility (Oomen et al., 2014) and is regulated by (early)stress-exposure and MR activation (Gass et al., 2000; Heine et al., 2004; Naninck et al., 2015). To assess the long-term effect of ELS on hippocampal neurogenesis depending on the genetic background of the animals, a different cohort of mice was generated to examine the levels of neurogenesis at 4 months of age. Neurogenesis was measured in the entire DG and also along both the suprapyramidal blade and the infrapyramidal blade of the hippocampus, since neurogenesis is not homogeneous in both blades and each might have distinct functions (Olariu et al., 2007; Sahay and Hen, 2007; Snyder et al., 2009).

For DCX positive cells (**Figure 5A**; typical example in **Figure 5D**), there was a significant interaction between genotype and ELS [*F*(1,31) = 6.892, *p* < 0.014] in the entire DG. *Post hoc* analysis revealed a significantly increased number of DCX positive cells in MR-tg mice exposed to ELS when compared to wildtype animals that were exposed to ELS (*p* < 0.012). Furthermore, MR-tg mice exposed to ELS displayed a trend toward increased DCX positive cells when compared to non-stressed MR-tg mice (*p* = 0.033). In the suprapyramidal blade, there was a significant interaction between genotype and ELS [*F*(1,31) = 5.153, *p* < 0.031]. Follow-up analysis showed a trend toward an increase in DCX positive cells in MR-tg stressed mice compared to ELS controls (*p* < 0.05). A significant interaction between genotype and ELS was also seen in the infrapyramidal blade [*F*(1,31) = 6.857, *p* < 0.014] with MR-tg ELS mice showing a trend toward an increased number of DCX positive cells compared to the wildtype ELS group (*p* = 0.024).

**FIGURE 5:** **Structural plasticity in MR-tg and control mice.** Bar graphs represents the averaged results for: **(A)** DCX positive cells, **(B)** Ki67 positive cells and **(C)** BrdU positive cells. For all markers, we analyzed the total number of positive cells in the whole DG and along the suprapyramidal (supra) and infrapyramidal blade (infra). Data are expressed as mean ± SEM with *p*-values based on *post hoc* LSD. *n* = 6–10 animals per group. ^∗^significant, *p* ≤ 0.0125. **(D)** Shows a representative image of DCX staining in the control group.

Analysis of Ki67 positive cells (**Figure 5B**) showed a significant main effect of genotype [*F*(1,31) = 25.040, *p* = 0.001] with an increase of Ki67 positive cells in MR-tg mice. This main effect was also seen In the suprapyramidal blade [*F*(1,31) = 33.747, *p* = 0.001] and the infrapyramidal blade [*F*(1,31) = 13.512, *p* = 0.001]. No significant effect of ELS nor an interaction effect between ELS and genotype were found in the total number of Ki67 positive cells or in the suprapyramidal and infrapyramidal blades.

With respect to the number of BrdU positive cells (**Figure 5C**), a significant main effect of ELS [*F*(1,31) = 5.301, *p* < 0.029] and of genotype [*F*(1,31) = 5.301, *p* < 0.029] was present in the entire DG, but no interaction effect. In the suprapyramidal blade, there was a significant main effect (increase) of ELS [*F*(1,31) = 5.419, *p* < 0.028]. In the infrapyramidal blade no significant overall effects were found.

### Electrophysiology

Since alterations in synaptic function underlie learning and memory processes, we examined mEPSCs, mIPSCs and evoked AMPA and NMDA currents after ELS and investigated whether effects were modified by overexpression of MRs. Electrophysiological recordings revealed an interaction effect between genotype and ELS for mEPSCs [*F*(1,41) = 4.333, *p* < 0.044] and for mIPSCs [*F*(1,41) = 6.263, *p* < 0.017] with regard to the frequency (**Figures 6A,B**; typical traces in **Figure 6E**). *Post hoc* analysis revealed no significant effects on the frequency of mIPSCs and mEPSCs between the experimental groups. No effects were present on the amplitude of the mEPSCs [*F*(1,41) = 0.080, *p* = 0.079, **Figure 6C**] and mIPSCs [*F*(1,41) = 0.880, *p* = 0.354, **Figure 6D**]. Similarly, the ratio between eEPSC/eIPSC [*F*(1,37) = 0.202, *p* = 0.656, **Table 1**] and the AMPA/NMDA ratio [*F*(1,34) = 0.008, *p* = 0.928, **Table 1**] was unaffected by ELS and/or MR overexpression. Finally, no effects of MR-tg or ELS were apparent on half maximal stimulus intensities and capacitance of granular cells in the DG (**Table 1**).

**FIGURE 6:** **Electrophysiological recordings in MR-tg and control (wildtype) mice, with or without early life stress (ELS). (A)** Effects on the frequency of **(A)** mEPSCs, and **(B)** mIPSCs, **(C)** amplitude of mEPSCs and **(D)** mIPSCs. Data are expressed as mean ± SEM, *n* = 11 cells per group. Traces **(E)** show typical examples of mEPSCs (top) and mIPSCs (bottom) recorded from a dentate granule cells at the holding potential mentioned at the right. Insets illustrate single events at a high time resolution.

**Table 1:** Capacitance of granule cells in the dentate gyrus (*n* = 11 per group); and half maximal stimulus intensity, eEPSC/eIPSC as well as AMPA/NMDA ratios (*n* = 8–10 cells per group).

	WT non-stressed	WT ELS	MR-tg non-stressed	MR-tg ELS
Capacitance (pF)	13.7 ± 1.3	12.8 ± 0.8	11.8 ± 1.1	14.8 ± 1.2
**Half maximal stimulus intensity(mA)**				
AMPA	0.87 ± 0.08	0.94 ± 0.09	1.00 ± 0.06	0.98 ± 0.12
GABA	0.77 ± 0.10	0.87 ± 0.12	0.81 ± 0.11	0.71 ± 0.05
**Ratios in evoked responses**				
eEPSC/eIPSC amplitude	0.72 ± 0.09	0.76 ± 0.09	0.91 ± 0.16	0.86 ± 0.11
AMPA/NMDA	29.9 ± 10.4	30.4 ± 11.0	40.0 ± 22.9	23.9 ± 6.3

*No significant interaction nor main effects were observed with respect to any of these parameters.*

## Discussion

Here we report that transgenic forebrain overexpression of MRs from postnatal day 15 (Lai et al., 2007) in mice alleviates the effects of ELS on non-stressful contextual memory formation at adult age. Moreover, we observed an interaction between ELS and MR overexpression on the number of DCX positive cells in the DG and the frequency of mEPSCs and mIPSCs in DG granule cells. These results suggest that MR overexpression may partly prevent or reverse ELS-induced changes in hippocampus-associated behavior as well as hippocampal structural and functional plasticity.

### Effects on Contextual/Spatial Memory

Our behavioral observations are in line with earlier studies showing that ELS hampers spatial memory formation tested under non-stressful conditions (Rice et al., 2008; Wang et al., 2013; Naninck et al., 2015). This is in agreement with other studies indicating that low levels of maternal care and maternal deprivation hamper spatial learning (Liu et al., 2000; Oomen et al., 2010).

While other studies have reported that low levels of maternal care and early life adversity enhance contextual fear memory formation (Champagne et al., 2008; Oomen et al., 2010) these effects were not found in our current study. Obviously, effects of early life adversity on the expression of contextual fear memory formation may depend on the ELS model that is used but also the testing paradigm in adulthood. Thus, in the same ELS paradigm we found that ELS results in enhanced expression of fear during cue-off periods in an auditory fear conditioning paradigm (Arp et al., 2016), indicating that ELS does impair the ability of animals to appreciate ‘safe’ moments in-between cue exposure.

Mineralocorticoid receptors play a critical role in learning and memory. During stress exposure, these receptors moderate the switch between spatial and stimulus-response strategies (Schwabe et al., 2010; Vogel et al., 2015). Moreover, mice with genetic ablation of MRs are impaired in spatial learning and contextual fear learning (Berger et al., 2006; Zhou et al., 2010). Importantly, our current results indicate that enhanced MR activation may overcome effects of ELS.

### Structural and Cellular Effects

To investigate the possible neurobiological substrate through which MRs may affect contextual memory in animals exposed to ELS, we examined neurogenesis and synaptic transmission in the DG, which are known to be important for spatial and contextual memory (Morris et al., 2003; Pastalkova et al., 2006; Whitlock et al., 2006; Kitamura et al., 2009). We did not observe effects of ELS *per se* on the number of DCX positive cells, Ki67 positive cells or on the survival (BrdU staining) of newborn cells. Similar observations in this ELS model have been reported before with this ELS model in mice (Naninck et al., 2015). Yet, we did see an interaction effect with regard to the number of DCX-positive cells, possibly related to the fact that MR-tg mice displayed increased numbers of DCX positive (and Ki67) positive cells, particularly after ELS. No effects were seen on the number of BrdU positive neurons in the DG. Thus, MR overexpression may enhance the generation and maturation of newborn cells in the DG, but not their survival.

Genetic deletion of MRs has been reported to reduce proliferation of new born cells in adult (but not in young) mice (Gass et al., 2000). This finding is in line with the current observation that overexpression of MRs enhances proliferation in the DG. Our observation that ELS enhances the number of DCX-positive cells specifically in MR-tg mice is more unexpected. Thus, enhanced proliferation –based on the result with Ki67 staining- in combination with (slightly) enhanced survival –as inferred from BrdU staining- were observed both in control and in ELS MR-tg mice. One possibility is that ELS regulates maturation of new born cells specifically in MR-tg animals. In support, some ELS models are known to alter hippocampal GR expression (reviewed in Anacker et al., 2014) and maturation of new born cells was earlier shown to depend on GR expression in the dentate (Fitzsimons et al., 2013); since GR and MR share their natural ligand corticosterone, changing the expression level of MR may affect that of GR, which could explain why the effect of ELS is particularly prominent in MR-tg mice. Alternatively, Ki67 and BrdU positive cells do not necessarily reflect only neuronal cells which makes the link between changes in Ki67 and BrdU labeling and changes in DCX+ cells not very precise. Future studies will need to identify whether changes in Ki67 labeling and BrdU labeling are present in neuronal cell types after ELS and in MR-tg animals. In addition, it will be interesting to investigate whether the increase in DCX+ cells is accompanied by increased dendritic complexity although we have no evidence that ELS or MR overexpression affects dendritic complexity in the hippocampal CA3 area (Kanatsou et al., 2015a) or hippocampal CA1 area (unpublished observations). At present, we found the strongest effects of ELS and MR-overexpression on DCX+ cells in the suprapyramidal blade. This may be behaviorally relevant given the notion that neurons in the suprapyramidal blade show greater experience-related activity and mature later than those in the infrapyramidal blade (Snyder et al., 2012).

In agreement with the effects on behavior and neurogenesis, we observed an interaction effect between ELS and MR overexpression on the frequency – but not amplitude – of mEPSCs and IPSCs. These results suggest that MR moderates effects of ELS on spontaneous synaptic transmission. However, it should be noted that for both experimental endpoints *post hoc* analysis did not reveal a significant effect of ELS in the wildtype animals, which differs from the observations in behavior. Also, neither the AMPA/NMDA ratio of evoked excitatory responses nor the ratio of evoked excitatory versus inhibitory responses were affected. This is somewhat unexpected, since earlier studies reported that these parameters may be sensitive to early life stress (Brunson et al., 2005; Bagot et al., 2012; Rodenas-Ruano et al., 2012).

In summary, human and animal studies suggest that enhanced MR function may confer resilience to stressors, and MR activation prevents hippocampal granular cells from apoptosis (Sloviter et al., 1989) and facilitates synaptic potentiation (Pavlides et al., 1994). Based on our current studies, it is tempting to speculate that enhanced neurogenesis and spontaneous synaptic transmission in MR overexpressing (compared to wildtype) mice may contribute to overcoming detrimental effects of ELS on spatial memory formation, but the cellular effects were rather modest and a causal relationship clearly awaits further investigation.

## Conclusion

Our data reveal that MR overexpression may confer resilience to the effects of stress exposure during early life on contextual memory formation. Comparable observations have been made for other mediators of the stress response such as CRH (Ivy et al., 2010; Wang et al., 2011).

Of interest, MR overexpression in the currently used model starts approximately at PND15 (J. R. Seckl, personal communication), i.e., after the period of ELS. Since it is not known at which point in time structural and functional properties of the hippocampus start to deviate, eventually resulting in behavioral deficits, it is currently difficult to judge whether MR overexpression reverses and normalizes deviations that have already started at PND15 or prevents the development of delayed effects induced by ELS. Regardless, the fact that changes in MR expression starting after ELS has taken place result in hippocampal function that is indistinguishable from that seen in non-stressed wildtypes has interesting translational potential. These studies may provide new avenues to interfere with vulnerability factors (such as CRH) or resilience factors (such as MR) to promote behavioral performance after early life adversity.

## Author Contributions

All authors were involved in writing and approving the manuscript. SK, HK, DK, RvdA, and JdB carried out the experiments. AH and JS generated the transgenic mice. HJK and MJ designed and supervised the study.

## Conflict of Interest Statement

The authors declare that the research was conducted in the absence of any commercial or financial relationships that could be construed as a potential conflict of interest. The reviewer SG and handling Editor declared their shared affiliation, and the handling Editor states that the process nevertheless met the standards of a fair and objective review.
